This article has been retracted.

# Intelligent Prediction and Optimization Algorithm for Chronic Disease Rehabilitation in Sports Using Big Data

**DOI:** 10.1155/2021/9920421

**Published:** 2021-04-30

**Authors:** Xuelei Zhang, Xiaofeng Wang

**Affiliations:** ^1^Physical Education Department, Institute of Disaster Prevention, Langfang 065201, Hebei, China; ^2^Sports Department of Hebei Vocational College of Rail Transportation, Shijiazhuang 050000, Hebei, China

## Abstract

This paper investigates chronic diseases in the older population in the Chinese province of Henan and analyzes the rehabilitation needs and the current supply of related services in different levels of medical and elderly care institutions. We explore the fundamental causes for the diversified needs and insufficient supply of chronic disease patients in professional medical services and daily care. Using big data and deep learning (DL) in the sports domain, we propose a novel and intelligent prediction system for chronic diseases. Our model explores effective sinking methods of high-quality medical resources, training and guidance practices, assistance and guidance measures, and the ability to improve the grassroots services so that more chronically ill populations can stay in the community family as long as possible. In such an environment, they can receive cheap, safe, and suitable services. It can also lead to further improvement in constructing the government's regional medical rehabilitation care service system and can formulate long-term care relevant compensation policies.

## 1. Introduction

The United Nations “Global Population Development Report” shows that, as of June 2015, the global population reached 7.3 billion. The report claims that about 12% are aged 60 and above, and it is growing at an annual rate of 3.26%. It is estimated that, by 2030, the elderly population will reach 1.4 billion, and by 2050, it will exceed 2 billion, which will account for 21% of the world's total population. The current global aging [1, 2] situation is severe and irreversible. In 2012, the death rate of residents from chronic diseases accounted for 86.6% of the total death rate, which includes cancer [3], cardiovascular [4] and cerebrovascular diseases [5], and chronic respiratory infections [6].

Noncommunicable diseases are often referred to as chronic diseases. Such diseases have the characteristics of long-term and sometimes hard to heal. The unpredictability that occurs and the sudden exposure of disease risks will cause economic, health, and psychological risks [7]. This type of chronic disease has long course characteristics, incurable and frequent comorbidities, and its severe epidemic situation. From a global perspective, the 2017 Global Burden of Disease Study released by The Lancet in 2018 showed that chronic diseases' mortality rate reached 73.4%. From 2007 to 2017, the total mortality rate caused by chronic diseases increased by 22.7%, and the disease burden increased rapidly. According to the latest public data, China has more than 300 million patients with chronic diseases [8]. In 2018, the number of deaths from chronic diseases accounted for 86.6% of the total domestic deaths.

In 2018, China's disease burden accounted for approximately 74% of chronic diseases. It is an enormous disease burden in China. Among them, cerebrovascular diseases, tumors, and chronic respiratory diseases, which cause death, accounted for the most considerable proportions. Among the chronic diseases, hypertension, diabetes, and chronic obstructive pulmonary disease are the three conditions with the heaviest disease burden [9]. Hypertension alone accounts for 25.2% of the total mortality rate, and the disease type diabetes accounts for 9.7 percent. The mortality rate caused by chronic obstructive pulmonary disease accounted for 9.9%, especially for the elderly. Using 2013 China's chronic disease and its risk monitoring data, it was found that more than three-quarters of Chinese elderly over 60 were suffering from chronic diseases. The coexistence of the characteristics of chronic diseases among the population is serious, and the prevalence is high. From the majority and mortality of chronic diseases in China in the past five years, chronic diseases' burden is still increasing. A priority-based strategy is required to deal with chronic diseases, and special attention should be paid to it. The precise positioning of this increasingly large number of vulnerable groups will help build a well-off society in an adaptable way [10]. Based on this current situation, the elderly patients with chronic diseases are selected as the research objects, aiming at health poverty vulnerability, which is currently not well explored. To do so, one must consider five levels of personal population characteristics, personal health status, medical security system, health service demand, and health behavior. Recent works [11, 12] examine the influencing factors of this issue to achieve the accuracy of key poverty alleviation targets, improve the protection mechanism of medical insurance, and truly solve the health poverty problem of elderly patients with chronic diseases.

With the rapid development of big data and deep learning (DL) technologies in recent years, we have a more scientific approach to tackle this problem. In this paper, we propose a new type of chronic disease intelligent prediction system. The proposed method makes use of big data and DL in the sports domain [13]. Our model explores high-quality medical resources, training, and guidance approaches and auxiliary guidance measures to improve grassroots services' level and ability to enable more chronically ill older people to live in communities or families for a long time. The model will also obtain cheap, safe, and suitable services, further improving regional medical care, rehabilitation, and elderly care [14] as a government service system. Long-term care policies provide a basis and reference for related compensation policies.

Following are the main contributions points of this paper:

1. Using big data and DL in the sports domain, this paper proposes a novel chronic disease intelligent prediction model, which can help formulate a scientific chronic disease rehabilitation plan.
2. To improve prediction accuracy, a dual network tracking hierarchical attention mechanism was proposed. First, we train and search for images of older people with chronic diseases through two branches. Then, we use a convolutional neural network to extract more robust features, enabling the target to obtain better tracking results under illumination changes and background interference conditions.
3. We also conducted simulation experiments. Experimental results show that the algorithm can effectively predict the development trend of chronic diseases in the elderly and give medical advice, helping formulate long-term care policies.

## 2. Background

### 2.1. Elderly Patients with Chronic Diseases

Chronic noncommunicable disease (NCD) having relatively hidden onset, complicated etiology and conditions, low awareness and control rate, prolonged illness, a longer course of medication, high disability, and mortality can cause serious harm to individuals, families, and society. These diseases mainly include endocrine system diseases (such as diabetes, hyperthyroidism, and hypothyroidism), cardiovascular and cerebrovascular diseases (such as stroke, hypertension, coronary heart disease, and acute myocardial infarction), chronic respiratory diseases (such as chronic obstructive pulmonary disease, chronic bronchitis, and asthma), malignant tumors, and oral diseases among others [15]. In developing countries, the standard for the elderly is 60 years old and above, and in developed countries, it is 65 years old and above.

### 2.2. Basic Characteristics of Elderly Patients with Chronic Diseases

The top 5 chronic diseases with prevalence are 225 cases (68.6%) of hypertension, 150 cases (45.7%) of osteoporosis, and 121 cases (36.9%) of coronary atherosclerotic heart disease. Besides, there were 113 cases of diabetes (35.1%) and 71 cases (21.6%) of chronic gastritis. The coexistence of chronic diseases and multiple diseases is up to 11%, with an average of 4.68 ± 1.96. Also, 7 patients with only one disease have 2.1% of chronic diseases [16]. The remaining 321 cases (97.9%) have multiple chronic diseases comorbid; the disease course is about 1–720 months, an average of 197.89 ± 149.08 months.

### 2.3. Artificial Neural Networks

Neural networks originated from the study of biological neurons. Inspired by this, researchers put forward the concept of artificial neurons, also called perceptrons. The neural network [10–14] model is composed of many neurons. Each neuron defines a new learning model, which receives input, processes it, and outputs accordingly [17]. As shown in Figure 1, after employing the weight and bias terms, the perceptron feeds the output to the activation function, which further generates a particular outcome.

*x*_1_, *x*_2_,…, *x*_*n*_ is the input unit of the neuron, which defines the input data, *w*_1_, *w*_2_,…, *w*_*n*_ is the weight coefficient responsible for processing the data, and then *b* is the bias term, and *y* is the output after processing through an activation function. Then the input model of the neuron can be expressed as follows:

(1) $$\begin{array}{c} V=\overset{n}{\underset{i=1}{\sum }}w_{i}x_{i}+b,\\ y=\varphi \left(V\right), \end{array}$$

where *φ*(*∗*) represents the activation function, which can be sigmoid, softmax, tanh, Relu, or Gelu. A generic neural network consists of three parts: the input layer, the output layer, and the middle's hidden layer [18]. Each layer will add bias and weight terms, where each hidden layer contains several neurons. Besides, under the nonlinear activation functions, the neural network can learn deeper content characteristics.

## 3. Objects and Methods

### 3.1. Research Objects

Using the multistage sampling method, we divide the province into 18 parts as per the administrative settings. According to the 2014 statistical data of the province, we also categorize the medical and health institutions of each city (first-level hospitals, community health service centers, the third-level hospitals, and the second-level hospitals that have been standardized and assessed by the health administrative department) and public elderly care institutions with more than 100 beds into five floors [19, 20]. Using the random number table method, we randomly select one from each of the five tertiary hospitals' levels, resulting in 90 hospitals. Then, 10 staff members were randomly selected from each institution, and 10 patients with chronic diseases from each institution, that is, a total of 900 staff members and 900 patients with chronic conditions, were surveyed.

#### 3.1.1. Service Organization Inclusion and Exclusion Criteria

1. Inclusion criteria: (a) we established first-level hospitals, second-level hospitals, third-level hospitals, and community health service centers according to the plan approved by the health administrative department following the former Ministry's hospital rating evaluation standards of health; and (b) elderly care institutions and public institutions directly under the civil affairs department and have more than 100 beds
2. Exclusion criteria: medical institutions and pension institutions that are fully invested or jointly built by companies, enterprises, and social capital

#### 3.1.2. Staff Inclusion and Exclusion Criteria

1. Inclusion criteria: (a) on-the-job professional and technical personnel, who have obtained corresponding practicing qualification certificates; (b) employment system staff, working on a full-time basis for more than 3 months; and (c) those who agree to participate in this survey voluntarily
2. Exclusion criteria: (a) during the investigation period, those who are not on duty due to rotation, going out, etc.; (b) the institution's non-in-service staff enrolled in advanced studies and internships; and (c) those who withdrew during the investigation period

#### 3.1.3. Inclusion and Exclusion Criteria for the Elderly with Chronic Diseases

1. Inclusion criteria: (a) age ≥60 years; (b) all chronic diseases have been diagnosed by medical institutions at the second level and above and meet the diagnostic criteria for various chronic diseases; (c) consciousness, normal cognitive function, able to communicate and effectively cooperate; and (d) those who give informed consent and voluntarily participated in the research
2. Exclusion criteria: (a) severe dysfunction of the heart, brain, liver, kidney, and other organs, who are in the acute or terminal stage of the disease; and (b) withdrawal during the investigation period

### 3.2. Dual Network Based on Hierarchical Attention Mechanism

Inspired by the deep neural networks, we use a dual network tracking framework of the layered attention mechanism. By introducing the attention layer to find the importance of each channel and then recalibrate these channels, the valuable features are strengthened, and features not related to the target are suppressed. Then, we use a fusion layer to combine the deep and shallow features to extract more detailed target information. Such an approach is more robust in complex situations (such as target occlusion and illumination changes). The model then responds to the feature response maps of different layers of the network. Then, we use the AdaBoost algorithm for the weighted integration to make significant errors get a smaller weight. The minor error gets a larger weight so that the filter with a more vital decision ability can play a crucial role.

#### 3.2.1. Dual Neural Network

As shown in Figure 2, the dual network has two inputs: one is the template *z* and the other is the search area *x*. The inputs {*z*, *x*} are then fed into two different neural networks, which process the input to a new space and a different representation. By learning a similarity function *f*(*z*, *x*), the model calculates the similarity between the template and finds the candidate block with the most prominent resemblance on the new picture as this article's target position. Generally, the template block is the input image in the first block. The advantage of the fully convolutional neural network is that the search area's image does not need to be the same size as the template image, and a larger search area image can be used as input. The similarity function can be expressed as follows:

(2) $$\begin{array}{c} f\left(z,x\right)=\phi \left(z\right)*\phi \left(x\right)+b_{1}, \end{array}$$

where *ϕ*(*z*) is a convolution kernel, convolved on *ϕ*(*x*), and *b*_1_ represents each position's value in the score map. This paper uses the discriminative method to train the positive and negative sheep of the search image. The target log loss can be defined as

(3) $$\begin{array}{c} l\left(y,v\right)=\log\left(1+\exp\left(-y*v\right)\right), \end{array}$$

where *y* represents the true value, ranging in (−1,1), *v* represents the actual score of the search image of sample one, the probability of a positive sample is (1/1+*e*^−*v*^), and the probability of a negative sample is 1 − 1/(1+*e*^−*v*^); then, the target training can be obtained by the definition of cross-entropy. The average log loss of all positions at the time is

(4) $$\begin{array}{c} L\left(y,v\right)=\frac{1}{D}\sum_{u\in D}l\left(y\left[u\right],v\left[u\right]\right), \end{array}$$

where *D* represents the final score map and *u* represents all positions in the score map. The trained convolution parameter *θ* is minimized by the stochastic gradient descent method to obtain the optimal solution:

(5) $$\begin{array}{c} \arg\underset{\theta }{\min}=\underset{\left(z,x,y\right)}{E}L\left(y,f\left(z,x;\theta \right)\right). \end{array}$$

The advantage of the dual network is that its network structure is divided into two branches, and it shares the parameters of the convolutional layer. As long as the network is trained on the training parameters, it is only a detection and matching task. The template frame it uses is the first frame of the image, and it will make the target not adaptable to changes in the environment. When the target undergoes massive deformation or external factors, the first frame of the image cannot learn more about the target. Features and only the center position of the target are obtained. When the scale of the target changes, a multiscale method is required to regress the target, which increases the amount of network calculation and reduces the speed and accuracy of tracking.

#### 3.2.2. Attention Mechanism

The visual attention mechanism is similar to the human brain [4–9] signal processing mechanism for vision. Humans can quickly scan what they see and quickly find the target area that needs attention. The focus of visual attention generally injects more observations into this area. You can notice the details of this target area information and then ignore useless information in other areas. The attention mechanism in deep learning [21–23] is similar to the human visual attention mechanism. It also selects essential information related to the target from a variety of image information [24, 25].

As shown in Figure 3, the image source elements are composed of a series of <Key, Value, and Query>. The first stage calculates the similarity or correlation between the query and each key by providing the search's target element value. Then, in the second stage, the first stage's value is normalized, and the weight coefficients corresponding to the value corresponding to each key can be obtained. Finally, the weighted sum of these weight coefficients can return the final attention value. The first stage introduces the cosine function to calculate the similarity between the query and each key value as follows:

(6) $$\begin{array}{c} \text{Similarity}\left(Q,K\right)=\frac{Q*K}{\left\|Q\right\|*\left\|K\right\|}. \end{array}$$

In the second stage, we use the softmax function to convert the first stage's result with a similarity score. The similarity value of the first stage can be normalized, and the weight of critical information can be emphasized through the softmax function, which is calculated as follows:

(7) $$\begin{array}{c} a_{i}=\text{Soft}\max\left({\text{sim}}_{i}\right)=\frac{e^{{\text{sim}}_{i}}}{\sum_{i=1}^{L_{x}}e^{{\text{sim}}_{i}}}, \end{array}$$

where *a*_*i*_ represents the weight of each Value_*i*_, *L*_*x*_=Source represents the length of the source, and finally, we perform a weighted sum of these weights to obtain the final attention value:

(8) $$\begin{array}{c} \text{Attention}=\left(Q,S\right)=\overset{L_{x}}{\underset{i=1}{\sum }}a_{i}*{\text{Value}}_{i}. \end{array}$$

The corresponding attention value can be obtained for each query. A small amount of helpful information can be filtered from a large amount of data information and focus on this valuable information, ignoring the most useless information.

### 3.3. Dual Network of Hierarchical Attention Mechanism

As shown in Figure 4, this section is based on the dual network framework to predict chronic diseases of the elderly. The network has two branches, one corresponding to the sample image branch, generally, the first frame image *Z*, and the other is the search image branch, the current frame image *X*.

The two images are trained through a convolutional neural network asynchronously. Then, after a series of operations, the sample image is relabeled with the feature map through the attention module, and then, the search image is related to the operation. Finally, we got a prediction result between the two; here, it is also applied to the layered features. Then, the model fuses the output prediction results on the third and fifth layers of the convolutional neural network and obtains the final target prediction result. The matching function between these two branches can be expressed as follows:

(9) $$\begin{array}{c} R^{n}=\underset{i}{\sum }\text{Conv}\left(\phi_{i}^{n}\left(Z\right),\phi_{i}^{n}\left(X\right)\right)+b. \end{array}$$

## 4. Experiments

### 4.1. Experimental Environment

Table 1 describes the experiment's hardware platform and software simulation environment settings used in the paper.

### 4.2. Training

We use stochastic gradient descent (SGD) to minimize the log loss when training the model from scratch. The training dataset uses the ILSVRC2015-VID dataset, which contains more than 30 basic categories and 4500 target image sequences for training. The initial value is set using Gaussian distribution, and the scale is set according to the improved Xavier method. The initial learning rate of the convolutional layer is set to 0.001. The training process includes 50 iterations, each iteration includes 5000 sample pairs, and the learning rate becomes 0.87 every 50 epochs.

### 4.3. Evaluation Method

To analyze the network performance, we use a confusion matrix-based evaluation strategy for our proposed model. We can intuitively understand how much data of a particular chronic disease in the test set is correctly predicted through the confusion matrix and how many chronic disorders are incorrectly predicted. The confusion matrix can be expressed as follows:

(10) $$\begin{array}{c} \text{ACC}=\frac{\text{TP}+\text{TN}}{\text{TP}+\text{TN}+\text{FP}+\text{FN}}. \end{array}$$

### 4.4. Experimental Results

With the intensification of aging, the number of older people with chronic diseases increases year by year. The surveyed subjects had 422 cases of two chronic diseases accounting for 48.51%, 203 cases of three chronic diseases accounted for 23.33%, 104 cases of four chronic diseases accounted for 11.95%, and 63 cases of five or more chronic diseases accounted for 7.24%. Some older people even suffer from 8 chronic diseases simultaneously, making it challenging to take care of daily housework by themselves, and going out activities are severely restricted. There are 34.25% of the elderly with chronic diseases who need to be cared for with different degrees of disability. This group's worries and clear cognition of health status are reflected in the results of health self-evaluation. The elderly who are diligent in fitness has the most negligible proportion of diseases, which shows that exercise is also essential for predicting chronic diseases. It can be seen from Table 2 that the algorithm in this paper has achieved good results in the prediction of various chronic diseases.

## 5. Conclusion

This paper investigates the chronic diseases of the elderly in Henan Province, China. It analyzes the content of medical and elderly institution's rehabilitation needs at all levels and the current status of related service providers. We proposed a dual network tracking algorithm based on a hierarchical attention mechanism. First, train and search the images of the elderly with chronic diseases through two branches, and then use the convolutional neural network to extract more robust features. The target can obtain better prediction results in complex environments for exploring the effectiveness of innovative, high-quality medical resources. Our model explores sinking methods, training and guidance methods, and auxiliary and guidance measures to effectively improve grassroots services' level and ability. A more chronically ill elderly can live in the community or family for a long time and can get cheap, safe, and suitable services. Furthermore, it improves the construction of regional medical care, rehabilitation, and elderly care, providing a basis for the government service system, formulating long-term care policies, and related compensation policies.

## Figures and Tables

**Figure 1:** Neuron structure diagram.

**Figure 2:** Proposed dual-path network framework.

**Figure 3:** Attention mechanism principle structure.

**Figure 4:** Dual network framework based on hierarchical attention mechanism.

**Table 1:** Experimental hardware platform and software simulation environment.

CPU	Intel (*R*) Core (TM) i5-8265U CPU @ 3.4 GHz
RAM	8.00 GB
Operating system	Windows 10
Development environment	PyCharm 2020.2.2
Programming language	Python 3.6.5

**Table 2:** The ACC (%) of different types of chronic diseases.

Type	ACC
Coronary heart disease	0.92
High blood pressure	0.96
Hyperlipidemia	0.95
Diabetes	0.93
Cataract	0.95
Asthma	0.92
Arthritis	0.94

## Data Availability

The data used to support the findings of this study are included within the article.
